# Cycloastragenol Confers Cerebral Protection after Subarachnoid Hemorrhage by Suppressing Oxidative Insults and Neuroinflammation via the SIRT1 Signaling Pathway

**DOI:** 10.1155/2022/3099409

**Published:** 2022-06-02

**Authors:** Weibin Lin, Hao Yao, Jinqing Lai, Yile Zeng, Xieli Guo, Shu Lin, Weipeng Hu, Junyan Chen, Xiangrong Chen

**Affiliations:** ^1^Department of Neurosurgery, The Second Affiliated Hospital of Fujian Medical University, Quanzhou, Fujian Province, China; ^2^Department of Neurosurgery, The Jinjiang Municipal Hospital, Quanzhou, Fujian Province, China; ^3^Centre of Neurological and Metabolic Research, The Second Affiliated Hospital of Fujian Medical University, Quanzhou, Fujian Province, China

## Abstract

Subarachnoid hemorrhage (SAH) is an acute cerebral vascular disease featured by oxidative insults and neuroinflammation. Cycloastragenol (CAG), the major active component of *Astragalus radix*, has a wide range of biological functions. However, the potential beneficial effects and the underlying molecular mechanisms of CAG on SAH remain obscure. In the current study, the cerebroprotective effects and mechanism of CAG on SAH were evaluated both in vivo and in vitro. Our results indicated that CAG significantly suppressed SAH-triggered oxidative insults, inflammatory mediators production, microglia activation, and the neutrophil infiltration in the brain. In addition, CAG improved neurological function and ameliorated neuronal apoptosis and degeneration after SAH. In vitro results also revealed the therapeutic effects of CAG on neurons and microglia co-culture system. Mechanistically, CAG treatment upregulated sirtuin 1 (SIRT1) expression, inhibited the levels of FoxO1, nuclear factor-kappa B, and p53 acetylation, and suppressed the subsequent oxidative, inflammatory, and apoptotic pathways. In contrast, inhibiting SIRT1 by pretreatment with Ex527 abrogated the protective actions of CAG both in vivo and in vitro models of SAH. Collectively, our findings indicated that CAG could be a promising and effective drug candidate for SAH.

## 1. Introduction

Subarachnoid hemorrhage (SAH) is a subtype of lethal stroke featured by high fatality and poor functional recovery. Although significant progress has been achieved to improve SAH outcomes, effective therapies for SAH are still lacking [1]. Recently, mounting evidence has indicated that early brain injury (EBI), characterized by inflammatory damage and robust oxidative insults, is the main cause of poor neurological outcome in SAH [2–6]. Theoretically, new therapies aimed at diminishing inflammation and oxidative stress would improve neurological outcome after SAH.

Sirtuin 1 (SIRT1), a member of the sirtuins family, exhibits a critical role in many biological processes, including oxidative stress, inflammatory response, aging, and energy homeostasis [7–9]. Emerging evidence has demonstrated that SIRT1 could protect against oxidative insults and inflammation in different research areas, such as ischemia reperfusion-induced renal, liver, brain, and heart injury [10–13]. In addition, the neuroprotective function of SIRT1 has emerged as a critical mechanism in a variety of central nervous system (CNS) diseases. In experimental SAH models, several studies have showed that SIRT1 is able to inhibit reactive oxygen species (ROS) generation, modulate microglia polarization, and ameliorate cerebral vasospasm [14–16]. All these suggest that SIRT1 could be a feasible target for treating SAH.

Astragalus radix, a traditional Chinese herbal medicine, has great potential for cardiovascular diseases, cerebrovascular diseases, diabetes, and cancers [17]. Cycloastragenol (CAG, Figure 1(a)) is the major active component of *Astragalus radix* [18]. Recent studies have demonstrated that CAG exhibits different biological actions including free-radical elimination, anti-inflammatory, and neurovascular protection activities [19–21]. More importantly, CAG could pass the blood-brain barrier and induce SIRT1 upregulation to ameliorate acute ischemic brain injury [18]. However, whether CAG is beneficial in SAH and the possible molecular mechanisms remain unknown. Therefore, we investigated the beneficial actions of CAG both in vivo and in vitro models of SAH and the underlying molecular mechanisms.

## 2. Materials and Methods

### 2.1. Experimental Animals

A total of 154 adult male Sprague-Dawley rats (230-260 g) were housed in standard conditions and were allowed to food and water freely. All experimental procedures were in accordance with the Guide for the Care and Use of Laboratory Animals of Fujian Medical University. Randomization of animals was conducted by using the website http://Randomization.com/.

### 2.2. In Vivo SAH Model

Rats were intraperitoneal injection with 1% sodium pentobarbital (50 mg/kg) before surgery. After anesthetization, a 4–0 monofilament nylon suture was inserted into the left internal carotid artery. After reaching the bifurcation of the anterior and middle cerebral arteries, the filament was advanced to puncture the artery [22]. Sham animals were treated via the same way except that vessel perforation. SAH hemorrhage severity score was evaluated by using an 18-point scoring system [23]. The sample taken for investigation is shown in Figure 1(b).

### 2.3. In Vivo Experimental Groups

In the first experiment, 91 rats were used. We divided animals into five groups: the vehicle-treated sham group (*n* =14), the vehicle-treated SAH group (*n* =21, 5 rats died), the 5 mg/kg CAG-treated SAH group (*n* =20, 4 rats died), the 10 mg/kg CAG-treated SAH group (*n* =18, 2 rats died), and the 20 mg/kg CAG-treated SAH group (*n* =18, 2 rats died). Postassessments included neurological functions, Nissl staining, and western blotting.

In the second experiment, 59 rats were used. We divided animals into four groups: the vehicle-treated sham group (*n* =12), the vehicle-treated SAH group (*n* =16, 4 rats died), the 10 mg/kg CAG-treated SAH group (*n* =15, 3 rats died), and the 10 mg/kg CAG plus Ex527-treated SAH group (*n* =16, 4 rats died). Postassessments included biochemical estimation, enzyme-linked immunosorbent assay (ELISA) assay, histopathological study, western blotting, and neurological functions.

### 2.4. In Vitro SAH Model

Haemoglobin- (Hb-) induced in vitro SAH model was performed according to a previous study [5]. For cell culture, the cortex was dissociated from rat pups (postnatal days 0-1). The primary cortical neurons and microglia co-culture system was maintained with Dulbecco's modified Eagle Medium with 10% fetal bovine serum. For SAH model in vitro, primary cells were incubated with 25 *μ*M Hb. The neuron-microglia co-cultures were assigned into control group, Hb + vehicle group, Hb +5 *μ*M CAG group, Hb +10 *μ*M CAG group, Hb +15 *μ*M CAG group, and Hb +15 *μ*M CAG + Ex527 group. Postassessments included cell viability analysis, biochemical estimation, enzyme-linked immunosorbent assay (ELISA), and immunofluorescence staining.

### 2.5. Drug Administration

For in vivo experiments, CAG (Yuanye Biotechnology, Shanghai, China) was dissolved in 5% DMSO (in saline). Different doses of CAG or vehicle were intraperitoneally administered at 3 h, 12 h, and then once daily for up to three days [18]. Ex527 (Sigma-Aldrich, St. Louis, MO) (10 mg/kg) or vehicle (1% DMSO) was intraperitoneally administered before SAH construction once daily for 3 days. For in vitro experiments, CAG was dissolved in culture medium. Ex527 (20 *μ*M in 1% DMSO) was applied for 24 h before Hb stimulation.

### 2.6. Cell Viability Evaluation

The Cytotoxicity Detection Kit (Roche) was performed in accordance with the manufacturer's protocols. Cell viability of each sample was determined at the wavelength of 490 nm using a spectrophotometer.

### 2.7. Intracellular ROS Generation

ROS Assay Kit (S0033, Beyotime, China) was employed to investigate ROS production. According to the manufacturer's protocols, the ROS content was measured by recording the mean relative fluorescence intensity.

### 2.8. Neurological Evaluation

As previously described, neurological deficit was calculated using a modified neurological severity score system. The low score indicated severe neurological deficits [23]. To further evaluate the motor impairments after SAH, the rotarod test was conducted. According to a previous report [24], rats were trained for 3 days before the formal testing. During the procedure, the latency to fall was recorded by investigators blinded to group information.

### 2.9. Western Blotting

Protein levels of ac-NF-кB, ac-FoxO1, SIRT1, and ac-p53 in brain samples were evaluated by western blotting according to standard protocols. In brief, the protein samples were blotted onto the PVDF membrane. Then, the membrane was incubated with primary antibodies against SIRT1 (Ab12193, 1 : 1000, Abcam), ac-FoxO1 (sc-49437, 1 : 200, Santa Cruz), ac-NF-кB (12629S, 1 : 500, Cell Signaling), ac-p53 (2570, 1 : 500, Cell Signaling), and appropriate secondary antibodies. *β*-Actin (BM0627, 1 : 4000, Boster Biotech) was the internal loading control for the proteins. Membranes were observed with enhanced chemiluminescence solution.

### 2.10. Immunofluorescence Staining

The brain sections and coverslips were fixed with 4% paraformaldehyde. Then, they were incubated in 0.1% Triton X-100 for 5 min. The slides were then incubated with primary antibodies including Iba-1 (SC-98468, 1 : 50, Santa Cruz), myeloperoxidase (MPO, SC-16128, 1 : 50, Santa Cruz), 8-hydroxydeoxyguanosine (8-OHdG, ab62623, 1 : 100, Abcam), SIRT1 (Ab12193, 1 : 100, Abcam), NeuN (MAB377, 1 : 200, EMD Millipore). After several times washes, they were incubated with appropriate secondary antibodies. The images were visualized by using an epifluorescence microscope.

### 2.11. TUNEL Staining

TUNEL staining was conducted by using a commercial kit (Roche Diagnostics, Indianapolis). The brain sections and coverslips were incubated with the reaction solution according to the instructions. The images were visualized by using an epifluorescence microscope.

### 2.12. Nissl Staining

In brief, brain sections were stained with Nissl solution for 10 min. After three times washing with PBS, they were sealed with neutral balsam. The damaged neurons had shrunken or contained vacuoles. The normal neurons had a relatively big and full soma, with round nuclei.

### 2.13. ELISA

After 24 h after SAH, animals were over-anesthetized. The supernatant samples from brain tissues were obtained. The levels of tumor necrosis factor-a (TNF-a), IL-6, IL-1*β*, and intercellular cell adhesion molecule-1 (ICAM-1) in tissue supernatant or culture medium were evaluated by using commercial ELISA assays.

### 2.14. Measurements of MDA, SOD, and CAT

After 24 h after SAH, animals were over-anesthetized. The supernatant samples from brain tissues were obtained. Commercial malondialdehyde (MDA) assay kit, superoxide dismutase (SOD) assay kit, and catalase (CAT) assay kit were used and the samples were evaluated as per the instructions.

### 2.15. Statistical Analysis

Results were expressed as the mean ± SD. One-way analysis of variance (ANOVA) test with Tukey's multiple comparison test was conducted. A value of *P* < 0.05 was considered significant. GraphPad Prism 8.02 was used for statistical analysis.

## 3. Results

### 3.1. Mortality

A total of 154 rats were used in our study, 4 rats with SAH grading score less than 8 were excluded. The mortality rate was 24.3% (9/37 rats) in the SAH + vehicle group; 15.5% (11/71 rats) in the CAG-treated SAH group; 25.0% (4/16 rats) in the SAH + CAG + Ex527 group. No rats died in the vehicle-treated sham group.

### 3.2. CAG Exerts a Beneficial Effect against SAH

As shown, western blotting results showed that CAG treatment at 10 and 20 mg/kg, but not 5 mg/kg, could significantly increase SIRT1 expression after SAH (Figures 1(c) and 1(d)). In addition, Nissl staining indicated that SAH insults induced overt morphologic changes and cellular degeneration, which could be ameliorated after different doses of CAG administration (Figure 1(e)). We further evaluated the behavior functions after SAH. It revealed that the functional deficits and motor function were severely impaired after SAH. In contrast, CAG treatment at 10 and 20 mg/kg could significantly reduce the neurological deficit scores and improve the time spent on the rotarod (Figures 1(f) and 1(g)). But CAG treatment at 5 mg/kg did not markedly make better functional behavior after SAH. No significant differences between 10 mg/kg and 20 mg/kg CAG treatment on neurological outcomes and SIRT1 expression were detected. These results revealed that CAG treatment at 10 mg/kg had the maximal protective effects after SAH. Thus, we used this dose in subsequent studies.

### 3.3. CAG Upregulated SIRT1 Expression and Reduced FoxO1, NF-кB, and p53 Acetylation after SAH

In the brain, SIRT1 is highly expressed in neurons and exerts an endogenous neuroprotection in many CNS diseases. As shown, western blotting data revealed that the expression of SIRT1 was further increased after CAG administration. Meanwhile, the acetylation levels of FoxO1, NF-кB, and p53 were effectively decreased in the SAH + CAG group as compared with SAH + vehicle group (Figures 2(a)–2(e)). Double immunofluorescent staining further confirmed that SIRT1 is mainly expressed in neurons post-SAH. In contrast, CAG further enhanced the expression of SIRT1 in neurons following SAH (Figures 2(f) and 2(g)). However, pretreatment with Ex527 abated the effects of CAG on SIRT1 expression as well as the subsequent SIRT1-mediated signaling pathway.

### 3.4. CAG Suppressed Inflammatory Response after SAH

Microglia activation, neutrophil infiltration, and the subsequent proinflammatory cytokines release play important roles in the neuroinflammation after SAH. We next evaluated the effects of CAG on neuroinflammation after SAH. As expected, SAH insults markedly raised the levels of IL-1*β*, TNF-a, IL-6, and ICAM-1 (Figures 3(a)–3(d)). In addition, SAH significantly induced microglia activation and neutrophil infiltration (Figures 3(e)–3(h)). In contrast, CAG supplementation effectively suppressed SAH-triggered microglia activation, neutrophil infiltration, and the proinflammatory cytokines production. But the anti-inflammatory effects of CAG on SAH were abated by Ex527 treatment (Figures 3(a)–3(h)).

### 3.5. CAG Inhibited Oxidative Insults after SAH

Next, we measured the antioxidant effects of CAG after SAH. 8-OHdG immunofluorescence staining confirmed that SAH aggravated oxidative insults (Figures 4(a) and 4(b)). Moreover, our data showed that SAH induced a significant increase in lipid peroxidation. In addition, the endogenous antioxidant enzymes including SOD and CAT were significantly suppressed after SAH insults (Figures 4(c)–4(e)). Treatment with CAG markedly reduced 8-OHdG immunoreactivity, decreased the content of MDA, and restored the impairment antioxidant systems. However, all these changes were counteracted by Ex527 (Figures 4(a)–4(e)).

### 3.6. CAG Inhibited Neuronal Apoptosis and Improved Neurological Function after SAH

Emerging evidence has shown that neuronal apoptosis is a key mechanism involved in neurological impairment after SAH. It revealed that SAH insults significantly aggravated behavior impairment. Moreover, TUNEL staining indicated that SAH insults induced a marked increase in neuronal apoptosis (Figures 5(a)–5(d)). In contrast, rats in the CAG-treated SAH group showed reduced percentage of apoptotic neurons and better neurological functions than rats in the SAH group. However, these changes were abated by SIRT1 inhibition with Ex527 (Figures 5(a)–5(d)).

### 3.7. CAG Ameliorated Hb-Stimulated Neuronal Damage

We further evaluated the effects of CAG on Hb-stimulated neurons and microglia co-culture system. A significant reduction in cell viability was observed in Hb-treated group. CAG treatment markedly improved cell viability after Hb stimulation in a dose-dependent manner (Figure 6(a)). In addition, Hb incubation triggered upregulations of inflammatory mediators (IL-1*β* and TNF-a) production, lipid peroxidation (MDA), and ROS production, all of which were diminished by CAG supplementation (Figures 6(b)–6(f)). In addition, CAG treatment markedly attenuated neuronal apoptosis after Hb stimulation. However, all the beneficial effects of CAG were abrogated by Ex527 treatment (Figures 6(a)–6(h)).

### 3.8. CAG Enhanced SIRT1 Expression In Vitro

We then measured the effects of CAG on SIRT1 expression in primary neurons. As shown, western blotting data revealed that the expression of SIRT1 was further increased after CAG administration (Figures 7(a) and 7(b)). In addition, compared to the Hb + vehicle group, SIRT1 immunoreactivity in primary neurons was further enhanced in the CAG-treated Hb group. These suggested that CAG could also upregulate SIRT1 expression in vitro (Figures 7(c) and 7(d)). In contrast, Ex527 abated the CAG-induced SIRT1 upregulation in primary neurons.

## 4. Discussion

This study verified that CAG protected against EBI after SAH both in vivo and in vitro. In vivo, CAG reduced SAH-triggered oxidative insults, inflammatory mediators production, microglia activation, and the neutrophil infiltration in the brain. In addition, CAG improved neurological function and ameliorated neuronal apoptosis and degeneration after SAH. In vitro, CAG also attenuated oxidative damage, inflammation, and neuronal cytotoxicity. All these actions of CAG were related with the upregulation of SIRT1 and the reduced acetylation of FoxO1-, NF-*κ*B-, and p53-mediated oxidative, inflammatory, and apoptotic pathways. In contrast, Ex527 inhibited SIRT1 expression and abated the neuroprotective effects of CAG after SAH. Thus, our data suggested that CAG attenuated SAH-induced EBI by activating of SIRT1-dependent pathway, and CAG might be a novel therapeutic drug for SAH treatment.

Accumulating evidence has revealed that oxidative damage and inflammatory response play critical roles in the pathogenesis of SAH [25–29]. Diminishing oxidative damage and inflammatory response could significantly improve neurological outcome after SAH [30–33]. CAG is the active form of *Astragalus Radix*, which exhibits a variety of pharmacological effects [18]. Previous studies have demonstrated that CAG could inhibit ROS production, ameliorate oxidative insults, and suppress inflammatory response in different disease models [17, 18]. However, the effect of CAG against SAH has yet to be investigated. In the current study, our data showed that SAH triggered a significant oxidative damage as evidenced by increased ROS production and decreased endogenous antioxidant activity. In addition, SAH markedly induced microglia activation, neutrophil infiltration, and proinflammatory cytokines release. Moreover, SAH insults resulted in evident neuronal death and neurological impairment. On the contrary, CAG treatment could significantly suppress oxidative insults and neuroinflammation after SAH. Meanwhile, CAG decreased neuronal apoptosis and improved functional outcomes in a SAH rat model. In vitro, CAG also dose-dependently ameliorated oxidative insults, inflammation, and neuronal damage. These suggest that CAG could protect against EBI after SAH by diminishing oxidative damage and neuroinflammation.

SIRT1, an NAD^+^-dependent class III histone deacetylase, exhibits a wide range of biological processes [34]. In the brain, SIRT1 is highly expressed in neurons and exerts an endogenous neuroprotection in a variety of neurological disorders [34–36]. Macarena et al. reported that SIRT1 protected the brain against cerebral ischemic damage by inhibition of neuroinflammation and apoptosis [35]. Zhou et al. suggested that activation of SIRT1 promoted mitochondrial biogenesis and reduced apoptosis after intracerebral hemorrhage [37]. In SAH, several studies have showed that activation of SIRT1 by pharmacological therapies could ameliorate neuroinflammation and oxidative insults, and improve motor functions [38–40]. In addition, SIRT1 has the potential to ameliorate cerebral vasospasm after SAH [14]. Whether CAG affects SIRT1 activation to exhibit neuroprotection after SAH remains obscure.

A previous study by Li et al. reported that CAG upregulated SIRT1-mediated signaling pathway and ameliorated brain injury in a middle cerebral artery occlusion mice model [18]. In agreement with this study, our data also showed that CAG significantly increased the expression of SIRT1 both in vivo and in vitro models of SAH. But how SIRT1 activation by CAG affects EBI after SAH remains unclear. As a histone deacetylase, SIRT1 could deacetylate a wide range of substrates [34]. In addition to histones, SIRT1 could deacetylate nonhistone protein substrates. For example, Sirt1 can target FoxO1 to protect cells from oxidative damage [41]. FoxO1 plays a key role in the maintenance of redox homeostasis. Overexpression of FoxO1 can induce endogenous antioxidant enzymes expression and enhance hydrogen peroxide scavenging [10]. Additionally, SIRT1 can deacetylate ly310 residue of RelA/p65 to downregulate NF-кB activity and inhibit proinflammatory mediators release [42]. Moreover, SIRT1 is able to deacetylate p53 to prevent the subsequent apoptosis [43]. Interestingly, our data revealed a significant increase in FoxO1, NF-кB, and p53 acetylation in the brain after SAH insults. In contrast, CAG upregulated SIRT1 expression and decreased FoxO1, NF-кB, and p53 acetylation after SAH. As a result, the oxidative stress, neuroinflammation, and neuronal apoptosis were all ameliorated by CAG treatment. To further confirm that SIRT1 has a beneficial role in the protective actions of CAG against SAH, we employed a selective SIRT1 inhibitor Ex527. As expected, Ex527 pretreatment inhibited SIRT1 expression, increased the acetylation of FoxO1, NF-кB, and p53, and abated the cerebroprotective effects of CAG against SAH. Therefore, our results strongly suggested that CAG could ameliorate EBI after SAH by upregulation of SIRT1-mediated neuroprotection.

Our study has several potential limitations. Firstly, some other targets of SIRT could be neuroprotective, for example, peroxisome proliferator-activated receptor-*γ* coactivator-1*α* and heat shock factor. Whether CAG could regulate these molecular targets after SAH remains unknown. Secondly, it is not convinced enough that activation of microglia is assessed only with iba1 staining. Other sensitive markers for microglia activation will be employed in our ongoing research. Thirdly, we did not evaluate the long-term effects of CAG after SAH. Moreover, although no side effects of CAG were reported, the pharmacokinetic studies are still required to validate the translational potential of CAG for SAH treatment.

## 5. Conclusion

Taken together, this study has identified that CAG notably ameliorated EBI after SAH by suppressing oxidative insults and neuroinflammation. The overall beneficial effects of CAG might involve in the SIRT1-dependent pathway. Our experimental results indicate that CAG may be a promising drug candidate for treating SAH.

## Figures and Tables

**Figure 1:** Dose-response effects of CAG on SAH. (a) The chemical structure of CAG. (b) Schematic representation of the cortex area sampled for evaluation. (c) Western blot analysis for SIRT1. (d) Quantification of protein expression of SIRT1 after CAG treatment (*n* =6 per group). (e) Representative photomicrographs of Nissl staining. Arrows point to degenerated neurons. Scale bar =50 *μ*m. Changes of (f) neurological deficits scores and (g) motor function after CAG treatment (*n* =9-10 per group). ^∗^*P* < 0.05.

**Figure 2:** Effects of CAG on SIRT1 signaling pathway. (a) Western blot analysis for SIRT1, ac-FoxO1, ac-NF-кB, and ac-p53. Quantification of protein expressions of SIRT1 (b), ac-FoxO1 (c), ac-NF-кB (d), and ac-p53 (e) after CAG treatment (*n* =6 per group). (f) Quantification of SIRT1 immunofluorescence staining after CAG treatment (*n* =6 per group). (g) Representative photomicrographs of immunofluorescence staining for SIRT1. Scale bar =50 *μ*m. ^∗^*P* < 0.05.

**Figure 3:** Influence of CAG on neuroinflammation after SAH. The levels of IL-1*β* (a), IL-6 (b), TNF-a (c), and ICAM-1 (d) were determined by ELISA assay (*n* =6 per group). (e) Immunostaining of Iba1 in brain sections. (f) Quantification of Iba1^+^ staining after CAG treatment (*n* =6 per group). (g) Immunostaining of MPO in brain sections. (h) Quantification of MPO^+^ staining after CAG treatment (*n* =6 per group). Scale bar =50 *μ*m. ^∗^*P* < 0.05.

**Figure 4:** Influence of CAG on oxidative damage after SAH. (a) Immunostaining of 8-OHdG in brain sections. (b) Quantification of 8-OHdG^+^ staining after CAG treatment (*n* =6 per group). Quantification of MDA (c), CAT (d), and SOD (e) after CAG treatment (*n* =6 per group). Scale bar =50 *μ*m. ^∗^*P* < 0.05.

**Figure 5:** Influence of CAG on behavior impairment and neuronal apoptosis following SAH. Changes of neurological deficits score (a) and motor performance (b) (*n* =12 per group). (c) Quantification of TUNEL^+^ staining after CAG treatment (*n* =6 per group). (d) Representative TUNEL images. Scale bar =50 *μ*m. ^∗^*P* < 0.05.

**Figure 6:** Influence of CAG on neuronal damage in vitro. Changes of cell viability (a), IL-1*β* (b), IL-6 (c), and MDA (d) after CAG treatment (*n* =6 per group). (e) Quantification of intracellular ROS expression after CAG treatment (*n* =6 per group). (f) Representative photomicrographs of immunofluorescence staining for ROS. (g) Representative photomicrographs of immunofluorescence staining for TUNEL. (h) Quantification of TUNEL^+^ neurons after CAG treatment (*n* =6 per group). Scale bar =50 *μ*m. ^∗^*P* < 0.05.

**Figure 7:** Influence of CAG on immunostaining of SIRT1 in vitro. (a) Western blot analysis for SIRT1. (b) Quantification of protein expressions of SIRT1 after CAG treatment (*n* =6 per group). (c) Representative microscopic images for SIRT1 immunostaining. (d) Quantification of SIRT1^+^ staining after CAG treatment (*n* =6 per group). Scale bar =50 *μ*m. ^∗^*P* < 0.05.

## Data Availability

The data that support the findings of this study are available from the corresponding author upon reasonable request.

## Abbreviations

8-OHdG: 8-Hydroxydeoxyguanosine
CAG: Cycloastragenol
CAT: Catalase
CNS: Central nervous system
EBI: Early brain injury
ELISA: Enzyme-linked immunosorbent assay
Hb: Haemoglobin
ICAM-1: Intercellular cell adhesion molecule-1
MDA: Malondialdehyde
MPO: Myeloperoxidase
ROS: Reactive oxygen species
SAH: Subarachnoid hemorrhage
SIRT1: Sirtuin 1
SOD: Superoxide assay dismutase
TNF-a: Tumor necrosis factor-a.
